# Reef-Fidelity and Migration of Tiger Sharks, *Galeocerdo cuvier,* across the Coral Sea

**DOI:** 10.1371/journal.pone.0083249

**Published:** 2014-01-08

**Authors:** Jonathan M. Werry, Serge Planes, Michael L. Berumen, Kate A. Lee, Camrin D. Braun, Eric Clua

**Affiliations:** 1 Australian Rivers Institute and School of Environment, Griffith University, Gold Coast, Queensland, Australia; 2 Ocean and Coast Research, Gold Coast, Queensland, Australia; 3 Centre de recherches insulaires et observatoire de l’environnement (CRIOBE), Moorea, French Polynesia; 4 Red Sea Research Center, King Abdullah University of Science and Technology, Thuwal, Saudi Arabia; 5 Biology Department, Woods Hole Oceanographic Department, Woods Hole, Massachusetts, United States of America; 6 Marine Mammal Research Group, Graduate School of Environment, Macquarie University, New South Wales, Australia; 7 Secretariat of the Pacific Community, CRISP Programme, Noumea, New Caledonia; 8 French ministry of Agriculture and Fisheries, Paris, France; University of California Davis, United States of America

## Abstract

Knowledge of the habitat use and migration patterns of large sharks is important for assessing the effectiveness of large predator Marine Protected Areas (MPAs), vulnerability to fisheries and environmental influences, and management of shark–human interactions. Here we compare movement, reef-fidelity, and ocean migration for tiger sharks, *Galeocerdo cuvier*, across the Coral Sea, with an emphasis on New Caledonia. Thirty-three tiger sharks (1.54 to 3.9 m total length) were tagged with passive acoustic transmitters and their localised movements monitored on receiver arrays in New Caledonia, the Chesterfield and Lord Howe Islands in the Coral Sea, and the east coast of Queensland, Australia. Satellite tags were also used to determine habitat use and movements among habitats across the Coral Sea. Sub-adults and one male adult tiger shark displayed year-round residency in the Chesterfields with two females tagged in the Chesterfields and detected on the Great Barrier Reef, Australia, after 591 and 842 days respectively. In coastal barrier reefs, tiger sharks were transient at acoustic arrays and each individual demonstrated a unique pattern of occurrence. From 2009 to 2013, fourteen sharks with satellite and acoustic tags undertook wide-ranging movements up to 1114 km across the Coral Sea with eight detected back on acoustic arrays up to 405 days after being tagged. Tiger sharks dove 1136 m and utilised three-dimensional activity spaces averaged at 2360 km^3^. The Chesterfield Islands appear to be important habitat for sub-adults and adult male tiger sharks. Management strategies need to consider the wide-ranging movements of large (sub-adult and adult) male and female tiger sharks at the individual level, whereas fidelity to specific coastal reefs may be consistent across groups of individuals. Coastal barrier reef MPAs, however, only afford brief protection for large tiger sharks, therefore determining the importance of other oceanic Coral Sea reefs should be a priority for future research.

## Introduction

Recent studies have highlighted the critical role that sharks play in regulating food chain diversity through top-down control [1], [2], [3]. In coral reef ecosystems, models suggest reduced reef resilience with shifts in coral to fleshy algal-dominated habitats possibly due to the absence of sharks and other predatory fish from coral reef systems [4], [5]. More recently, Sandin *et al*. [6] used underwater visual censuses at reef sites with different densities of top predators to show that fish species targeted by sharks tended to allocate more energy to reproduction than to somatic storage. This phenomenon led to increased biomass because of more individuals in spite of their smaller size compared to sites without sharks.

Unfortunately shark populations are declining on a global scale, largely due to illegal and uncontrolled fishing practises [7], [1]. This has led to concerns about shark populations in the Oceania region [8]. Overfishing and poaching are driven by an increasing demand for fins in the booming Asian economies [9]. Consequently, there is a critical need to support shark conservation through a better understanding of their ecology to insure the balance and long-term resilience of marine ecosystems [10]. This global conservation goal may be achieved using tools such as Marine Protected Areas (MPAs) at several spatial scales [11]. The declaration of MPAs can slow shark population declines [12], but the spatial scale must encompass the home range of the relevant species [13]. The extent of movement within and among high value coral reef habitats can vary with shark species, as some species are relatively sedentary (e.g. the blacktip, *Carcharhinus melanopterus*) [14] and others migratory (e.g. the tiger shark, *Galeocerdo cuvier*) [15]. These potentially complex movements can determine the role sharks play as trophic links between distant coral reef habitats, the potential interaction with fishing activities and the vulnerability of sharks to these pressures [16], [17], [18]. Therefore, identifying the movement patterns and habitat-use of key tropical shark species is essential for their conservation.

Many sharks undertake migrations and utilise resources in different habitats with site-fidelity varying at different spatial and temporal scales. This can influence the trophic role of larger predators in connecting distant habitats and reduce the risk of regional extinctions [19]. Furthermore, adults of species previously considered to exhibit strong reef fidelity (e.g. Grey reef whaler, *Carcharhinus amblyrhynchos*) have been shown to range further than previously thought, reducing the effectiveness of protected areas for these species [18]. As a first step, MPAs for top-level predators require an understanding of the spatial movements of individual sharks, the determination of centres of shark activity, the proportion of time spent in potential management areas and their migration pathways to and from these areas. In addition, ontogenetic differences need to be considered as many large sharks display increasing home ranges with size and maturity [13], [18], [20]. Heightened public concern about the occurrence of large and dangerous sharks in New Caledonian waters has arisen as a result of several human deaths since 2007 [21]. This makes it increasingly important to understand the localised and migratory movements of large sharks and how often they utilize regions with high human activity. A better understanding of the movement patterns of these migratory top predators is therefore essential, and the absence of ecological data is often a limiting factor for the efficacy of marine managed areas [22].

Despite the ecological importance of large species of shark and their direct and indirect influence on the distribution of prey and other species, information on the movements of large sharks has largely been confined to USA, Europe, South Africa and Australia [23]. In contrast, little is known about the movement of large sharks in New Caledonia and the Coral Sea. This is due to their wide-ranging, elusive behaviour and the challenges associated with their capture [12], [24]. Moreover, the development of better capture techniques and satellite and acoustic tagging technology has led to substantial advances in documenting the movements of these animals than was previously possible with traditional tagging techniques (e.g. [25]).

The tiger shark is one of the top-level predators in coral reef ecosystems and is listed as ‘near-threatened’ by the IUCN [26], [27]. It has a cosmopolitan distribution and occurs throughout the South Pacific, including the Coral Sea [28], [29]. Tiger sharks are often considered to be a reef-associated ‘coastal’ species that exhibits seasonal and diel visits to coral reef lagoons when traversing between coral shoals and atolls [30] and visits to areas with large prey items, such as green turtle, *Chelonia mydas*, rookeries (e.g. Raine Island, northern Great Barrier Reef, GBR), are independent of the prey’s nesting aggregations [31]. Tiger sharks provide important trophic links between distant habitats [32] and exhibit movements up to 6747 km, identified by conventional tagging [25], [33]. Directional movements occur across ocean basins [34], [35], during which dives to depths of 335 and 680 m have been documented via acoustic and satellite telemetry, respectively [34], [36]. Acoustic telemetry studies in Hawaii suggest tiger sharks occupy home ranges of at least 109 km of contiguous coastline with detections on acoustic receivers typically brief (mean = 3.3 mins) and interspersed by weeks, months and years [36]. In contrast, home ranges were considered to be larger but undefined by a study in Shark Bay, Western Australia, because satellite tracked tiger sharks displayed relatively low displacement rates relative to sharks tracked over shorter time periods [35]. Furthermore, in the Atlantic, satellite telemetry revealed that large female tiger sharks spent substantially more time in the open ocean rather than coastal areas, with long-range migrations confirming that this species is oceanic. These authors suggest, however, that patterns of reef residency and migration may vary for different sites, locations and regions around the world [37]. Recent work by Papastamatiou *et al*. [15] suggests the complexity of tiger shark movements could be due to triennial migrations of adult female tiger sharks triggered by their reproductive cycle. In addition to these observations, Driggers *et al.* [38] suggest it is probable that parturition occurs in shelf areas of less than 100 m deep where neonates remain until their first large-scale migration, as they found no areas of increased juvenile abundance associated with oceanic areas of high productivity. Importantly, the movements and habitat-use of tiger sharks, remain largely unknown in the Southwest Pacific.

The Coral Sea is a vast tropical/sub-tropical region in the Southwest Pacific comprising both significant coral reef systems around its boundary and open oceanic habitat with sea mounts and reef aggregations across its basin [39], [40]. Connectivity of reefs across the Coral Sea relies on sparse seamounts and reef aggregations, both in the Australian and French Exclusive Economic Zones (EEZ) [41]. Recent work suggest that these isolated seamounts, such as the Osprey and Shark reefs in the Australian EEZ, require urgent protection in order to conserve reef-associated shark populations [42]. Moreover, demonstrated interactions between large sharks and commercial long-lining and illegal shark-fining occur across the Coral Sea [41]. Despite this, information on the movement of large sharks in coastal coral reefs and open oceanic and seamount habitats in the Coral Sea is scant and as such the protection of large sharks in this region is of concern, particularly for wide ranging species that undertake large scale movements. Furthermore, recent work suggests the economic value of an individual shark is substantially greater when it is kept alive and available for various ecotourism activities [37], [43].

In March 2010 and affirmed in January 2012, a “declaration of intention between France and Australia for the Coral Sea sustainable management” was signed by the Minister for Foreign and European Affairs of the French Republic and the Minister for Foreign Affairs of the Commonwealth of Australia [44]. This document identified strategies for cooperative management of Coral Sea coastal and high seas ecosystems. Given the critical role of large sharks in this region, the future co-management process requires reliable ecological information for tiger sharks. The study we present herein sought to provide the type of information needed for effective management in the region. In the present study we used multiple tagging techniques to quantify the spatial dynamics of tiger sharks in the Coral Sea, with a particular emphasis on New Caledonia. The aims of this study were to (1) determine the level of site-fidelity to specific coral reef habitats and temporal connectivity (days to years) among habitats, (2) quantify the range of variation in movement patterns among individual tiger sharks and, (3) determine the extent to which these movement patterns represent migratory behaviours. In so doing we test the hypothesis that tiger sharks undertake regular or predictable migrations across the Coral Sea between New Caledonia and Australia with no difference in the habitat-use and site-fidelity at coastal barrier reefs of New Caledonia and Australia compared to oceanic reefs in the Coral Sea.

## Materials and Methods

### Ethics Statement

This research was done in accordance with permit No. 6024-4916/DENV/SMer (New Caledonia), permit No. G10 33187.2 (Great Barrier Reef Marine Park Authority), permit No. 143005 (Queensland Fisheries), permit No. QS2010 GS065 (Great Sandy Marine Park) and permit No. LHIMP/R/2012/009 (Lord Howe Island). This study was specifically approved by Griffith University ethics ENV/16/08/AEC. Sharks were also satellite tagged in Queensland (QLD) under Ocean and Coast Research animal ethics approval CA 2010/11/482.

### Study Area

The Coral Sea lies off the northeast coast of Australia (QLD) and is bounded in the east by New Caledonia, in the north by the southern extremity of the Solomon Islands and the south coast of eastern New Guinea (Fig. 1). On the western seaboard of this region and at similar latitudes along the tropic of Capricorn, the largest barrier reef system in the world (the Great Barrier Reef -GBR) extends along the east coast of Australia. Approximately 1000 km to the east, New Caledonia boasts the world’s second largest lagoonal reef system.

**Figure 1:** Seamounts and surrounding bathymetry across the Coral Sea between New Caledonia and Australia. Acoustic receiver array locations are shown along the east coast of Queensland, Australia and the southern Great Barrier Reef and inserts. Different shades of blue in the legend indicate different water depths.

Our study area included six key locations widely separated (>500 km each apart) to enable sampling and detection of shark movements across the spatial extent of New Caledonia, the Coral Sea and the east coast of Australia (Fig. 1): (1) Prony Bay in the south of New Caledonia, (2) Reef barrier off Belep archipelago in the north of New Caledonia, (3) the Chesterfield Islands in the centre of the Coral Sea, (4) Lord Howe Island in the central south of the Coral Sea, (5) Noosa to Rockhampton in Australia and (6) Mackay and Cairns in the central and far north of the GBR. New Caledonia has a large coral reef lagoon with interspersed island and barrier reefs separated by channels typically 30–40 m deep. The main island is surrounded by deep drop-offs to >1200 m with ocean basins separating the Loyalty Islands to the east and the Chesterfield Islands in the centre of the Coral Sea (Fig. 1). In the north of New Caledonia, Belep is lightly populated by local indigenous communities and is approximately 500 km to the north of Noumea, the capital of New Caledonia. Prony Bay in the south is approximately 100 km south of Noumea. A substantial nickel mine is situated near the bay and supports a working population of up to 10,000 people. From the west coast of New Caledonia a deep oceanic ridge runs south to the Lord Howe rise. To the west, Lord Howe basin (average 1500 m deep) separates the Chesterfields from the east coast of Australia. The Chesterfield Islands were used for commercial whaling in the early 1960s, but have been uninhabited by humans for over 40 years. This seamount sustains vast seabird populations and nesting green turtles. Isolated from Australia to the west and New Caledonian to the east by 500 nautical miles in either direction, the Chesterfield Islands lie at the northern end of a series of seamounts that run south in the centre of the Coral Sea to Lord Howe Island. On the east coast of Australia, the GBR extends from the north of Fraser Island to the northern tip of Queensland. Beyond the barrier reef the Australian continental plate extends out into the Coral Sea basin. We divided our capture, tagging and tracking efforts among these study locations (Fig. 1).

### Acoustic Tags

All but one of the captured sharks were tagged with acoustic transmitters via surgical implantation (see below). Acoustic transmitters, Vemco V16 R-coded 69 kHz acoustic tags (Amirix Systems Inc., Nova Scotia, Canada), were used to provide high-resolution movement information in key study areas and long-term measurements of site fidelity. Acoustic tag battery lives were estimated to be 696, 835, or 1448 days according to manufacturer specifications/estimates and differences in battery size, given a delay period of 50 to 130, 40 to 80, 30 to 90 s, respectively. Given average coastal sea-conditions, wind-strengths of 11–16 knots (20–29 km/hr), and high (H) or low (L) tag power output at 69 kHz, we assumed acoustic detection ranges of 400–800 m (www.vemco.com/education/range.php).

### VR2W Acoustic Receiver Arrays

Transmissions from these tags were detected by acoustic receivers moored underwater when a tagged shark came within acoustic range. Thirty Vemco VR2W acoustic receivers (Amirix Systems Inc., Nova Scotia, Canada) were deployed to passively track movements of tiger sharks from January 2009 to February 2013 (Fig. 1). Receivers were deployed in six separate arrays in (1) Prony Bay in the southern lagoon of New Caledonia 2009 (n = 8; Fig. 1A), (2) the barrier reef off Belep in the northern lagoon of New Caledonia in January 2010 (n = 3; Fig. 1B), (3) the Chesterfield Islands in the centre of the Coral Sea in August 2010 (n = 7; Fig. 1C), (4) Lord Howe Island in June 2012 (n = 4; Fig. 1D) and (5) receivers were also deployed in coastal areas along the east coast of Queensland, Australia, as part of the QLD Large Shark Tagging Program (QLSTP) (http://www.oc-research.com/pages/tagging-program.php) in March 2010 on the Sunshine coast (n = 4) and coastal area of Bundaberg to Rockhampton (n = 2), and (6) Mackay and Cairns (n = 2) in the GBR. Receivers on Lady Elliot Island, GBR, deployed by independent researchers studying Manta rays, Heron and One Tree Island, GBR, by the Australian Acoustic Tagging and Monitoring System (AATAMS) and Bourail, New Caledonia, by the Aquarium des Lagons and Université de la Nouvelle-Calédonie were also used to detect shark movements. One receiver deployed at Estree Pass in Belep in March 2010 received no detections and was subsequently relocated to Yande Passe, Belep, in August 2010. However, this receiver was unable to be retrieved in 2012 and was presumed missing. Receivers were moored on concrete filled tyres (as per Otway and Ellis [45]) in depths of 5–25 m or attached to anchored float lines approximately 5 m above the sea floor. Data were downloaded periodically throughout the study.

### Satellite Tags

We used two types of satellite tags: (1) Pop-up Satellite Archival Tags (PSATs) (models: MK10-PAT, miniPAT and Fastloc MK10-AF, Wildlife Computers, Redmond, WA, USA) to quantify swimming depths and migration pathways, and (2) dorsal fin-mounted, position-only satellite tags (SPOT5, Wildlife Computers, Redmond, WA, USA) to provide information on shark movements outside the detection range of our acoustic receivers.

### Geolocation of Satellite Tags

PSAT tags were pre-programmed to detach from the tiger shark 100–290 days after deployment. PSAT tags archived temperature, depth and light intensity data during deployment and transmitted to the Argos satellite array after the tags released from the shark. Light-based geolocations were approximated using proprietary software provided by the tag manufacturer (WC-GPE: Global Position Estimator Program suite, Wildlife Computers, Redmond, WA, USA) that employs threshold light-level geolocation methods [46]. Most probable tracks were constructed from these estimates using a state space unscented Kalman filter and blended sea surface temperature in the UKFSST library [47] for the R Statistical Environment [48]. Secondary bathymetric correction was performed using maximum daily depth of each individual in the analyzepsat library for R [49], [50] and 95% confidence interval envelopes were included in plots to illustrate the equivalent error bubble around most probable tracks. Due to lack of approximated locations from WC-GPE, the most probable track for one individual (TS 25) was constructed using raw light levels in a state space model performed in the TrackIt library for R [51] followed by bathymetric correction.

SPOT tags transmit a signal to the Argos satellite array whenever the dorsal fin breaks the surface for long enough (i.e. 15 to 30 seconds). This provides a near real-time estimate of the shark’s position. The accuracy of the position estimate however, depends on the number and time between transmissions received during a satellite pass and are classified as either 3 (<250 m), 2, (250–500 m), 1 (500–1,500 m) and 0, A or B (1,500 to 3000 km) [52]. Z positions provide no estimates of the shark’s position. We used all class 3, 2 and 1 positions to plot tracks and included class 0, A or B positions if these were within a realistic swimming distance at a maximum speed of 3.5 km hr^−1^ [34], [53] from a previous class 1–3 position, capture location or acoustic receiver detection.

### Shark Capture and Tagging Procedures

At each location large sharks were captured using barbless hook and line (baited with tuna pieces) and restrained in a specially designed harness developed by Werry *et al*. [54] (Fig. 2). Captured sharks were guided into the harness, which was placed parallel to the vessel. The restrained shark was maintained with its head directed into the current to ensure constant flow of water over the gills. Sharks were then tail-roped and inverted to initiate tonic immobility. Sharks remained docile in this position while morphometrics of total length (TL) (cm) and gender were recorded. Dorsal fins and distinguishing body features of all captured sharks and tiger sharks that broke away from baited lines before tagging were photographed as per Clua *et al.* [55]. The harness also enabled the opportunistic identification of stomach contents for sharks that regurgitated their contents after capture and restraint in the harness. For individual comparisons, tiger sharks were assigned ontogenetic categories of mature, sub-adult or juvenile. Size-at-maturity estimates of 330 cm TL and 292 cm TL for females and males respectively were determined based on tiger sharks from Hawaii [56]. The presence of semi-calcified claspers were used to define sub-adult males and sharks >259 cm TL for sub-adult females. Juveniles were defined as <259 cm TL for females and the presence of non-calcified claspers for males. A Vemco R-code V16 transmitter was then surgically implanted into the body cavity through a small incision in the abdominal wall (as per Holland *et al.* [34]). PSAT tags were attached to selected tiger sharks by creating a small incision in the shark’s skin at the base of the dorsal fin and inserting a titanium dart under the skin. The titanium dart was then locked in place with a small stitch. SPOT tags were attached on selected sharks by creating 4 small holes near the top of the shark’s dorsal fin and using threaded nylon with washers and lock nuts to secure the tag. After tagging, sharks were maintained in the harness while the research vessel slowly moved forward to push oxygenated water over the gills of the shark. Tagging and capture stress was monitored as per Werry *et al*. [54]. Sharks swam away vigorously on release (Video S1), although one tiger shark in the Chesterfields was also released via underwater assistance on scuba.

**Figure 2:** Restraint of 3.8 m tiger shark in harness.

### Behavioural Patterns

Localised behavioural patterns of tiger sharks with acoustic tags were defined into four categories. (1) Passer-by, for individuals never detected on acoustic arrays after the first month of release after acoustic tagging. (2) Transient, for individuals that were re-detected on individual acoustic arrays after temporal periods greater than one month. (3) Pseudo-Resident, for individuals detected on the same acoustic array for more than five days within each month for three or more months of the year and for <30% of their potential detection period, and (4) Residents, for individuals detected within ten or more months in each year within individual acoustic arrays and for >30% of their entire potential detection period.

### Statistical Analysis

Data from receivers were processed to define the length of time an individual was monitored (calculated as release date till date of last detection), the number of days an individual was present during the monitoring period, the average number of days between subsequent detections, the movements within and between acoustic arrays and the difference in diel detection frequency. Significant differences in proportion of detections between night (18∶00 to 5∶59, sunset to sunrise) and day (6∶00 to 17∶59, sunrise to sunset) detected between individuals were determined using Chi-square. A standardized Residency Index (RI) was calculated for all sharks as the total number of days a tiger shark was detected within an acoustic receiver array divided by the number of days the shark could possibly have been detected assuming its transmitter worked for the period of estimated battery life [57].

To determine if there were differences in the space use of each of the satellite tagged sharks three-dimensional 50% and 95% kernel utilisation distributions were calculated using methods described in Simpfendorfer *et al*. [58] using the ‘ks’ package in R [59]. This method incorporates both horizontal and vertical movements together to provide a more accurate representation of the shark’s movement [58]. The plug-in bandwidth was used to calculate smoothing factor for the kernel estimation as it has been shown to be the most appropriate for bandwidth for home-range studies (see [60]). No further statistical analysis was conducted on the 3D kernels due to the high variability in the number of days that each shark was tracked.

## Results

### Characteristics of Acoustic and Satellite Tagged Sharks

Thirty-four tiger sharks 154–390 cm TL were captured across five study locations between October 2008 and October 2012 (Table 1). Thirty-three sharks were tagged with acoustic transmitters: four males and six females in the Southern Province of New Caledonia, one male and three females in Belep, Northern New Caledonia, four male and six females in Chesterfield and eight females and one male on the east coast of Australia. Tiger sharks on the east coast of Australia were tagged with acoustic tags as part of the QLSTP. Female tiger sharks were primarily sub-adult (n = 10). Fewer adult females were captured (n = 4), of which only one was captured and tagged within New Caledonia. Juvenile sharks (n = 4) were captured only in the Southern Province while both sub-adult (n = 2) and mature (n = 4) males were captured in the north and south of New Caledonia and at the Chesterfield Islands in the centre of the Coral Sea. Only a single male was tagged within the Australian study locations.

**Table 1:** Tiger sharks monitored at New Caledonia (Southern Province, Northern Province), the east coast of Australia (Southern Queensland and the Great Barrier Reef) and the Chesterfields in the Coral Sea with acoustic tags.

TigerShark	TaggingLocation	Date ofCapture	Sex	TL(cm)	days bwtagging andfirst detection	No. ofdaysmonitored	No ofdaysdetected	No. ofdetections	Av minutesat eachstation	Max lineardistance bwdetections (km)
1	SP	30/01/2009	F	154	192	1273	14	39	4.5	5.5
2	SP	7/07/2009	F	164	10	1141	6	55	5.7	3.5
**3**	SP	1/02/2010	F	192	na	906	0	0	0	–
4	SP	9/07/2009	F	270	21	1143	9	35	6.75	6.75
5+	SP	1/10/2008	F	300	495	–	–	–	–	1442
**6**	SP	26/01/2009	F	300	0	1277	1	1	1	0.9
7	SP	13/07/2009	M#	312	0	1139	1	2	4	0.9
**8**	SP	13/07/2009	M*	340	0	1139	3	8	2.5	2
**9**	SP	24/08/2010	F	370	225	702	31	91	3.14	5.5
10	SP	28/01/2009	M*	380	62	1275	30	103	4.35	10.9
**11**	SP	15/07/2009	M*	390	405	875	2	20	1.3	4.7
12	NP	4/03/2010	F	286	200	875	1	2	1	1
**13**	NP	4/03/2010	F	290	110	875	5	31	4	1
**14**	NP	11/03/2010	M#	294	267	868	1	3	3	244
15	NP	3/03/2010	F	338	28	876	7	11	2.85	1
**16**	CI	12/08/2010	F	260	6	432	155	872	4.13	22
**17**	CI	13/08/2010	F	270	2	432	36	438	12.2	0
**18**	CI	12/08/2010	F	310	4	595	255(4)	2948(68)	5.5	22(742)
19	CI	16/08/2010	M*	310	8	432	183	1292	3.93	22
20	CI	18/11/2011	M*	323	YBR					
21	CI	25/11/2011	M*	323	YBR					
22	CI	20/11/2011	M*	328	YBR					
23	CI	22/11/2011	F	329	YBR					
24	CI	12/08/2010	F	330	13	432	2	10	6	14.4
**25**	CI	15/08/2010	F	332	14	858	3(1)	9(9)	2.5	9.5(761)
26	C GBR	20/04/2011	F	232	YBR					
27	C GBR	20/04/2011	F	260	YBR					
28	C GBR	20/04/2011	F	276	YBR					
**29**	C GBR	31/10/2012	M*	346	YBR					
**30**	C GBR	30/10/2012	F	367	YBR					
**31**	C GBR	31/10/2012	F	370	YBR					
32	SQ	1/03/2011	F	210	YBR					
33	SQ	21/09/2011	F	270	YBR					
34	SQ	19/09/2011	F	300	98	98	1	2	2	117

Individual sharks bolded and underlined were also tagged with various satellite tags (see Table 2).

+refers to shark identified with photo-ID.

refers to mature males.

^#^ refers to male sharks with semi-calcified claspers. TL refers to total length. Tagging locations include, SP (Southern Province, New Caledonia), NP (Northern Province, New Caledonia), CI (Chesterfields), SQ (Southern Queensland, Australia), C GBR (Cairns, Great Barrier Reef).

–indicates no data available. na refers to not applicable. YBR refers to yet to be recorded. Brackets for TS18, TS 25 refer to detections on the GBR.

Of these sharks, fourteen were also tagged with satellite tags (Table 2), three with SPOT tags and 11 with PSATs. Sharks with acoustic tags were detected over total days (d) ranging from one to 255 (less than the battery length of the acoustic tags)(median 4.5 d) with two to 858 days between acoustic tagging and first detection on either an array closest to location of tagging or another array in the study location (median 28 d)(Table 1). This compared to detection periods of four to 210 days (median 19 d) for PSATs and seven to 38 days (median 13 d) for SPOT tags (Table 2). With the exception of TS9, TS11 and TS29, premature release occurred for all PSATs, and no data was received from two PSAT tags deployed in Australia on mature females (Table 2).

**Table 2:** Tiger sharks monitored at New Caledonia (Southern Province, Northern Province), the Chesterfields in the Coral Sea and Cairns (GBR) with satellite tags.

TigerShark	TaggingLocation	Sex	TL(cm)	Satellitetag typeand id	MK10Pop-off date,SPOT 5 lasttransmission	Duration ofdeployment(days)	Max distancefrom releasepoint (km)	Max depthduringdeployment(m)	Modaldepth(m)	Meandepth(m)	Maxtemp(°C)	Mintemp(°C)	Modaltemp(°C)	Meantemp(°C)
3	SP	F	192	SPOT 5	11/03/2010	38	240	–	–	–	–	–	–	–
6	SP	F	300	MK10	2/02/2009	4	208	80	64.0	48.5	26.2	25.1	26.1	25.7
8	SP	M*	340	MK10	1/08/2009	19	150	368	40.0	53.0	24.4	14.4	23.8	23.2
9	SP	F	370	MK10	22/02/2011	181	1141	1136	16.0	11.2	26.2	5.6	22.0	**–**
11	SP	M*	390	MK10	11/02/2010	210	154	640	40.0	61.0	28.8	8.2	23.7	23.5
13	NP	F	290	SPOT 5	17/03/2010	13	60	–	–	–	–	–	–	–
14	NP	M#	294	SPOT 5	17/03/2010	7	23	–	–	–	–	–	–	–
16	CI	F	260	miniMK10	27/08/2010	15	124	312	62.5	55.0	24.4	17.8	23.6	23.0
17	CI	F	270	Fast-locMK10	17/08/2010	4	–	19	12.0	13.9	27.8	22.8	23.6	23.7
18	CI	F	310	miniMK10	13/12/2010	93	207	536	39.5	91.0	27.4	9.4	24.0	20.7
25	CI	F	332	Fast-locMK10	22/08/2010	7	101	66	40.5	28.0	32.2	23.4	23.6	23.8
29	C GBR	M*	346	MK10	31/10/2012	78	240							
30	C GBR	F	367	Fast-locMK10	30/10/2012	DNR								
31	C GBR	F	370	Fast-locMK10	31/10/2012	DNR								

Tiger shark numbers correspond to sharks with acoustic tags in Table 1.

refers to mature males.

^#^ refers to male sharks with semi-calcified claspers. TL refers to total length. DNR refers to did not report.

### Acoustic Monitoring

Patterns of acoustic detections differed between acoustic arrays and individuals. Individual temporal patterns of occurrence were highly variable in coastal arrays and displayed little evidence of residency (Fig. 3, 4), however sharks tagged in 2010 and monitored until November 2011 in the Chesterfield Islands, with the exception of mature females, displayed consistent patterns of movement and strong residency (Fig. 3, 4). These individuals undertook extensive excursions between receivers within the array area in the Chesterfields with continual movement patterns back and forward across the lagoon that varied with each individual (Fig. 5). Days detected for these sharks ranged from 36 to 255 across all months of the year (Fig. 5). In contrast, the number of days tiger sharks were detected on acoustic receivers in the Southern Province varied from 0 to 31 with one mature 370 cm TL female (TS9) and a mature 380 cm TL male (TS10) displaying pseudo-residency behaviour (Fig. 6). Days detected for tiger sharks varied between one to seven in Belep and zero to one in Australia.

**Figure 3:** Temporal occurrence of tiger sharks tagged at New Caledonia (Southern Province, Belep), the southern GBR and the Chesterfield Islands in the Coral Sea with acoustic tags. Individual sharks are numbered with sex (M = male; F = female) (see Table 1) and arranged by increasing body size from top to bottom within each study location. Numbers are bolded for mature sharks. Note shark 34 F was tagged at Fraser Island (Australia) and 14 M was detected at Bourail (New Caledonia) after being tagged at Yande Pass (Table 1). χ refers to tagging date. Blue dots indicate detections in the respective acoustic arrays. Δ refers to end of available reception period for an acoustic array or tag.

**Figure 4:** Residency Index (RI) of tiger sharks tagged at New Caledonia, the southern GBR and the Chesterfield Islands in the Coral Sea with acoustic tags. Individual sharks are numbered (see Table 1) and arranged by increasing body size from top to bottom for those tagged in the Coral Sea (top section) and those in New Caledonia/GBR (bottom section). Numbers are bolded and sex (M = male; F = female) shown for mature sharks.

**Figure 5:** Spatial occurrence of tiger sharks tagged at the Chesterfield Islands in the Coral Sea with acoustic tags. Individual tiger shark numbers correspond to Table 1. Arrows indicate direction of movement between receivers; double headed arrows indicate repeated movements between receivers. Coloured bubbles indicate the proportion of detections at numbered acoustic receivers. Shades of blue in the legend are labelled to indicate different water depths. Inset bar graphs indicate the number of days detected in each month and localised behaviours; PB (Passer-by), T (Transient), PR (Pseudo-Resident), R (Resident). Blue arrows indicate the month of capture.

**Figure 6:** Spatial Occurrence of tiger sharks within the Southern Province (A to H) and Northern Province (I) monitoring arrays in New Caledonia (see Fig. 1). Individual tiger shark numbers correspond to Table 1. Arrows indicate direction of movement between receivers; double headed arrows indicate repeated movements between receivers. Coloured bubbles indicate the proportion of detections at numbered acoustic receivers. Different shades of blue in the legend indicate different water depths. Inset bar graphs indicate the number of days detected in each month and localised behaviours; PB (Passer-by), T (Transient), PR (Pseudo-Resident), R (Resident). Bar graph arrows indicate the month of capture. Numbers alongside the bubbles correspond to receiver number.

Mature females (TS24 and TS25) in the Chesterfield Islands, however, were detected for only two and three days respectively and exhibited similar patterns of transitory and asynchronous occurrence to those of tiger sharks detected in coastal acoustic arrays (Fig. 3, 4 and 5). More than half of the sharks detected on acoustic arrays displayed transitory or a combination of pseudo-residency and transitory behaviour, with the remaining eight sharks detected in coastal arrays displaying passer-by behaviour (Table. 1, Fig. 4 and 6). For example, TS34 was briefly detected once, 117 km from her tagging location off Fraser Island, Australia, by an acoustic receiver at Lady Elliot Island (Fig. 7). Likewise, TS14 tagged at Yande Pass, Belep, was detected at Bourail, New Caledonia, on an acoustic receiver array deployed by another research team over 240 km from the shark’s tagging location (Table 1; Fig. 7). In addition TS25 was detected at One Tree Island, adjacent to Heron Island on the GBR 842 days after being tagged in the Chesterfields in August 2010. Furthermore, TS18 was detected at Lady Elliot Island, GBR, 591 days after being tagged in the Chesterfields in August 2010 and at Heron Island, GBR, 595 days after being tagged. This shark displayed strong residency to the Chesterfields for her first year of tracking before detection on the GBR. Both TS 18 and TS 25 displayed migrations of over 600 linear km providing direct evidence of temporal connectivity between oceanic reefs of the Coral Sea in New Caledonia and the GBR. All tiger sharks were detected only on acoustic receivers closest to their respective capture locations except TS14, TS18, TS25 and TS34. Tiger sharks were detected across all months in the south of New Caledonia irrespective of ontogeny or sex (Fig. 3, 6). Movements between acoustic receiver stations in the Southern Province occurred primarily in the Woodin Channel and the coral bommie in the greater lagoon. One 380 cm TL mature male (TS10) was detected well within Prony Bay at the Carenage River on several occasions. Visits at individual stations were typically brief as sharks were typically detected only once within a three minute period on individual stations. No tiger sharks were captured, tagged or detected at Lord Howe Island during the period of acoustic receiver deployment.

**Figure 7:** Spatial patterns of tiger shark movements across the Coral Sea between 2008 and 2013. Bubble plots show 95% confidence interval envelope for PSAT tracks. (A) Satellite tracks of PSAT tiger sharks tagged in the Southern lagoon of New Caledonia; (B) SPOT satellite tagged tiger sharks in the north of New Caledonia; (C) PSAT tiger sharks in the Chesterfield Islands, and (D) off Cairns in the GBR. (E) Includes the straight distance between the first photo-ID spotting of TS5 in New Caledonia and the second on the east coast of Australia. (F) The movement of a juvenile TS in the south of New Caledonia. Red arrows indicate movements from point of release to detection on spatially separated array for tiger sharks with acoustic tags. Orange arrows indicate generalised patterns/directions of major currents within the region of tiger shark migration. EAC refers to the East Australian Current.

Overall 55% of the 33 tiger sharks with acoustic tags were detected after release. 30% were yet to be recorded (detected) (YBR) and one shark was resighted although this shark was not tagged (Table 1). Diel patterns of detection showed individual differences between day and night for sharks detected for sufficient temporal periods (Table 3).

**Table 3:** Diel patterns of tiger shark occurrence at acoustic receiver stations.

TigerShark	TaggingLocation	Date ofCapture	Sex	TL (cm)	day timedetections	night timedetections	X^2^	P
1	SP	30/01/2009	F	154	30	9	19.4	<0.001
2	SP	7/07/2009	F	164	5	50	34.2	<0.001
4	SP	9/07/2009	F	270	20	15	7.7	0.398
9	SP	24/08/2010	F	370	56	35	24.3	0.028
10	SP	28/01/2009	M*	380	44	58	14.6	0.166
16	CI	12/08/2010	F	260	474	389	173.4	0.004
17	CI	13/08/2010	F	270	62	374	203.2	<0.001
18	CI	12/08/2010	F	310	1081	1868	443.7	<0.001
19	CI	16/08/2010	M*	310	526	522	175.8	0.902

Chi-square analysis and P values refer to day and night time detections.

### SPOT Tracks

Three tiger sharks fitted with SPOT tags produced 43 positional fixes between February and March 2010. Most of these positions (n = 34) were from TS3, a 192 cm TL juvenile tagged in the Southern Province. Interestingly, TS3 was not detected on any of the acoustic receivers in the vicinity of her tag and release location, however SPOT positions showed she moved throughout the Southern Province, remaining within the lagoon and adjacent to the barrier reef for the period of her tracking (Fig. 7). Alternatively, TS13 (n = 7) and TS14 (n = 2) had few positional fixes, although TS13 was periodically redetected on acoustic receiver stations at her original tagging location after 200 days. TS14 was also detected on another acoustic array after 294 days (Table 1).

### PSAT Tracks and Ocean Migration

Eight tiger sharks fitted with PSATs revealed long distance, open-ocean and inter-island migrations with seven of these sharks detected on acoustic arrays at the site of capture after four to 405 days (Fig. 7). Tiger sharks tagged in the Southern Province showed migrations out of the main lagoon into open-ocean. TS6 moved south and was one of two satellite tagged sharks in New Caledonia not to be detected on an acoustic receiver. TS8 migrated east towards the Loyalty Islands, whereas TS11 migrated into the Coral Sea south of New Caledonia before returning to the Southern lagoon after 210 days. During this journey, TS11 underwent dives of up to 640 m. TS9 underwent a significant migration south and appeared to be oriented to the oceanic Norfolk ridge. TS9 spent most of her time near the surface, but underwent a deep dive of 1136 m to waters of 5.6°C (Fig. 8C). This shark then moved south past Norfolk Island before turning north back along the Norfolk ridge. TS9 was then detected back on the southern New Caledonia acoustic array after 225 days (Fig. 7).

**Figure 8:** Depth-temperature profiles of selected PSAT tagged tiger sharks. (A) TS25 Chesterfield Islands, (B) TS11 South lagoon of New Caledonia, and (C) TS9 South Lagoon of New Caledonia. Black bars above A refer to periods of acoustic detection in the Chesterfield array. Note differing spatial and temporal scales.

Tiger sharks satellite tagged in the Chesterfield Islands showed movements out into open-ocean before returning to the lagoon and were then detected on the acoustic array. TS16 and TS17 appeared to be resident or pseudo-resident, whereas TS24 and TS25 were detected back on the Chesterfield array after 326 and 86 days, respectively. TS18 was tracked for 93 days. Interestingly, this shark showed numerous deep dives between periods of remaining at depths of no more than 40 m (Fig. 8A). Only one satellite tagged shark in the Great Barrier Reef (TS 29) provided a track for 78 days out into the Coral Sea off Cairns before the satellite tag popped-off west of Lizard Island. Satellite tags from two female tiger sharks 367 and 370 cm TL (Table 2) tagged in Cairns did not report (Table 2). Photo-ID of the dorsal fin of TS5 revealed the movement of this shark across the Coral Sea between Woodin Channel, Southern New Caledonia, in 2008 to Noosa Heads, Australia, in 2010 (Fig. 9). The combination of satellite and acoustic telemetry revealed the ocean migration and periodic return of TS11 to Woodin Channel 405 days after tagging.

**Figure 9:** Resightings of individual tiger shark based on dorsal fins. Arrows highlight the distinguishing features of the individual sharks fin. Note A1 was identified by Clua *et al*. [55]. The photo taken in A3 is after a tissue sample was taken from the second notch in the shark’s dorsal fin.

### Dive Profiles and Three-dimensional Habitat-use

Dive profiles showed extraordinary levels of vertical movement with the deepest depth on record for a tiger shark at 1136 m (Fig. 8). Three-dimensional 95% kernel estimates demonstrated tiger sharks utilised deep open ocean relatively close to the GBR, off Cairns (Fig. 10), whereas kernels suggest utilisation of the shallow lagoon with interspersed diving/movement down into deep water (possibly foraging) before returning to the lagoon. This pattern ties in nicely with the acoustic data (Fig. 3 and 8). The kernel estimates for the south of New Caledonia reflected the migration of sharks away from the southern New Caledonia lagoon, but indicated that the sharks also utilise the lagoon itself, which is a vast area with depths up to 80 m (Fig. 7F). Three-dimensional activity spaces (95%) averaged at 2.36×10^3^ km^3^ and varied from 0.16 to 4.48×10^3^ km^3^. Kernel estimates 50% varied from 37.7 to 9.49×10^2^ km^3^.

**Figure 10:** Individual 3D (95%) activity space of satellite tagged tiger sharks in the Coral Sea. (A) South New Caledonia: Green TS 6, Orange TS 8, Grey TS 11, (B) Chesterfields: Blue TS 16, Green TS 18, (C) Cairns: Purple TS 29.

### Patterns of Coral Reef Site-fidelity

Our study demonstrates extraordinary reef fidelity among tiger sharks in New Caledonia and the Chesterfield reefs. In New Caledonia, dorsal fin photo-ID of TS5 confirmed this shark was present in Prony Bay, New Caledonia, in 2002 on a whale carcass [55] and in 2008. As far as we are aware, this is the longest confirmed record of site-fidelity for a large tiger shark. This shark was later captured on shark control equipment at Noosa on the east coast of Queensland, Australia, in 2010 before being tagged and released by another research team (Fig. 9). In addition, TS 11 was captured and tagged with satellite and acoustic tags in New Caledonia in 2009 before returning to the site of capture in 2010. Eight sharks with satellite and acoustic tags were detected back on acoustic arrays at sites of release two to 405 days after tagging (median 24.5 d).

## Discussion

Tiger sharks monitored by a combination of acoustic and satellite telemetry across the Coral Sea utilised a remarkable range of habitat both horizontally among shallow coastal and island reefs and open ocean as well as vertically through the epi-, meso- and bathypelagic layers. This range of habitat-use is entirely consistent with results from previous studies conducted in other geographic regions (e.g. [34], [35], [36], [37]). The novelty in our findings is the remarkable year round residency of the sub-adult females and an adult male tiger shark in the isolated oceanic Chesterfield Island reef(s). Our study, however, did not support the hypothesis that tiger sharks undertake regular or predictable migrations between New Caledonia and Australia across the Coral Sea. Unlike other large apex predators and top level consumers, such as the white shark (*Carcharodon carcharias*) and humpback whale (*Megaptera novaeangliae*) which do appear to undertake consistent seasonal migrations within the Coral Sea (e.g. [61], [62], [63]), tiger sharks in our study displayed complex individual variability in both their wide-ranging migrations and localised movement patterns. Our results suggest discrete groups of tiger sharks across the Coral Sea utilise specific coral reefs incorporating nearby deep water oceanic environments 98 to 249 km from the location of tagging with three-dimensional (combined horizontal and vertical) activity spaces typically ranging from 0.16 to 4.48×10^3^ km^3^. In addition, our data suggest that selected individuals then undertake more wide-ranging migrations that provide temporal (but unpredictable and irregular) connectivity between reefs of New Caledonia and Australia. Recent work by Papastamatiou *et al.* [15] suggests this may be due to a phenomenon known as ‘partial migrations’ based on analysis of tiger shark movements in the Hawaiian island chain where only a proportion of the shark population migrate in a given period. In light of our data we propose two provisional and interlinked hypotheses related to mating/pupping and coastal vs oceanic reef-use to explain the observed migratory patterns.

### Mating/Pupping as a Driver for Adult Movement

Mature females were captured at all sites other than Lord Howe Island (LHI), although a small juvenile was filmed in 30 m of water on the LHI plateau during Baited Remote Underwater Video (BRUV) surveys undertaken by I. Kerr (LHI marine parks) providing evidence of pupping and the presence of mature females at this oceanic Coral Sea island (see Video S2). Mature females also displayed the longest migrations (e.g. TS9) and least frequent occurrence on acoustic receiver arrays suggesting they may be the main participants in wide-ranging movements that provide important temporal connections between ‘local’ groups of spatially separated (i.e. 500 km ) tiger sharks.

Mature females have triennial reproductive cycles [56] that probably drive unpredictable and seemingly inconsistent, yet extremely important, long-range migrations between mating and foraging grounds and suitable pupping habitats. Mating and pupping requirements may partially explain adult tiger shark migration patterns in the Coral Sea. Using random walk models from male and female tiger sharks recoded via passive acoustic telemetry in the Hawaiian Islands, Papastamatiou *et al.* [15] proposed that inter-island movements by tiger sharks were a result of a combination of partial reproductive migrations and individual decisions related to water temperature and primary productivity. This was also based on the limited inter-island movement of large males compared to that of mature females. Our data seemingly fit the proposed model of Papastamatiou *et al.* [15] and suggest that mature females may be of primary concern for conservation of tiger shark populations in the Coral Sea. For example, the transient nature of mature females in the Chesterfields compared to sub-adult and mature male sharks supports the notion that large females may move in three year cycles between pupping and foraging grounds on the east coast of Australia and the west coast of New Caledonia with mating taking place in the oceanic reefs in the Coral Sea. This strategy provides a largely unpredictable means of utilising sparse foraging and pupping habitats, but increased and varied mating opportunities with males that may be more restricted in their movements. Isotope analysis of tiger shark tissues from different regions in the Coral Sea will be a useful means to compare the signatures of males and females to further quantify these patterns [64]. In addition, blood analysis of adult females in coastal and oceanic areas will help to elucidate movements in response to parturition. This method was also proposed by Hammerschlag *et al*. [37] for tiger sharks in the Atlantic and Papastamatiou *et al.* [15] for tiger sharks in the Hawaiian Islands.

Our longest satellite track was undertaken by a 3.7 m female (TS 9) who undertook a directional migration of 1141 km from the coastal areas of the southern province of New Caledonia to close to Norfolk Island before being detected back at her coastal site of tagging after 225 days. During our survey efforts and repeat tagging trip in the Chesterfield Islands, we did not capture or observe small juvenile or new born tiger sharks; however, small juveniles were caught in the coastal areas (<60 m of water) of New Caledonia and have been recorded in Australia [65]. In addition, pregnant females have been recorded on the east coast of Australia, suggesting parturition occurs in these coastal areas.

Overall, general migration patterns of tiger sharks in the Coral Sea may be masked by highly variable individual movement patterns. In our study mature males showed high levels of site fidelity at oceanic reefs (e.g. TS 19) and repeated occurrence in only one of our defined tiger shark ‘group’ areas of the south of New Caledonia (e.g. TS 10), consistent with the model proposed by Papastamatiou *et al*. [15]. However, one male made a long range movement 294 km south along the west coast of New Caledonia, whereas TS 5 (a 3 m sub-adult female) showed extensive movement from southern New Caledonia to Noosa Heads, Australia, over a period of 495 days. TS 5 occurred in southern New Caledonia in 2002 and 2008 prior to its occurrence in Australia in 2010 (Fig. 9). In the future, new and advanced satellite tags (e.g. satellite-linked radio-telemetry (SLRT) tag with a multi-year battery capacity), such as those used over a two-year period by Domeier and Nasby-Lucas [66] on white sharks, may better reveal these movement patterns for large female tiger sharks.

### Localised Habitat-use

Our data lead us to reject our hypothesis of no difference in localised habitat-use of reefs across the Coral Sea by tiger sharks. In fact, we found an obvious difference in the shark behaviour between coastal (New Caledonia and GBR) and isolated oceanic reefs (Chesterfields). While we acknowledge differences in the number of receivers providing coverage in acoustic arrays, the novelty in our findings is the remarkable year round residency of the sub-adult females and an adult male tiger shark in the isolated oceanic Chesterfield reef(s). Satellite telemetry revealed members of this group of sharks made frequent deep dives, but acoustic data revealed frequent returns to the lagoon area with ongoing “patrolling” movements between cays across the lagoon. While Meyer *et a*l. [36] and Lowe *et al*. [30] demonstrate that isolated lagoons are important to Hawaiian tiger sharks and some individuals occur year round, we are not aware of any studies that have demonstrated year round, continual residency for large tiger sharks to the extent of those in our study.

Mature male and female tiger sharks utilise coastal and oceanic reef habitats in different ways most likely driven by a combination of female parturition requirements, suitable pupping grounds for offspring [56], [67] and utilisation of productive prey patches. Differences in female and male occurrence and habitat-use patterns have been recorded for other shark species, e.g. the oceanic short-fin mako, *Isurus oxyrinchus*, and blue shark, *Prionace glauca* [68] and coastal species such as the blacktip, *Carcharhinus melanopterus* [69] and scalloped hammerhead, *Sphyrna lewini* [70], [71] and were attributed to female avoidance of males as a strategy to increase fitness and reduce competition, different dietary requirements, and the locating of suitable pupping grounds for offspring [68], [70]. In our study area, data based on capture of 328 mature tigers in the QLD Shark Control Program between 2002 and 2012 along the QLD coast confirm the regular occurrence of both mature male and female tiger sharks (at a ratio of 1∶1.5). While adult male and female tiger sharks occur at sites across the Coral Sea, different life history requirements for males and females are likely driving individual differences in shark behaviour and habitat-use on both local and basin-wide scales in the Coral Sea.

### Coastal vs Oceanic Reef Foraging Hypothesis

Different reefs have varying prey and habitat characteristics that influence shark behaviour. The abundance and diversity of suitable prey available in the Chesterfields lagoon, in contrast to the sparsely distributed resources found on coastal reefs, may explain tiger shark residency. The Chesterfield reefs sustain large turtle populations including seasonal aggregations of breeding green turtles, populations of numerous sea snake species and breeding colonies of different species of sea bird (>200,000 individuals) in addition to teleost populations [41], [72]. For example, the stomach contents of one tiger shark (TS 19) tagged in the Chesterfield Islands contained hawksbill turtle (*Eretmochelys imbricata*), seabird and sea snake remains; prey items consistent with prey availability in the Chesterfields. Individual prey species do not necessarily explain residency as tiger sharks in the remote northern GBR do not necessarily occur in conjunction with the seasonal aggregations of the world’s largest breeding colony of green turtles at Raine Island [31]. However, Hawaiian tiger sharks undertake pelagic migrations between islands to coincide with seasonal prey accessibility such as the availability of fledging black-footed albatross, *Phoebastria nigripes* [32]. These anomalies around the Pacific Ocean add to the confusing and seemingly unpredictable patterns of tiger shark movement. However, the diversity of food resources and temporal variability in prey in the Chesterfields could explain the abnormally long residency (and absence of seasonality) of one adult male tiger in our study (TS 19) and indicates the Chesterfields may be a very important feeding ground for tiger sharks. In turn these favourable conditions may facilitate this area as a fertile mating ground. In contrast, adult female tiger sharks appeared to simultaneously leave the Chesterfields and were only briefly re-detected approximately one year after initial tagging, suggesting transitory behaviour among the isolated oceanic coral reefs probably due to the aforementioned mating/pupping hypotheses. Tiger sharks are true generalists and able to utilise wide and varied food sources and probably adapt their behaviour accordingly and with opportunity [73]. Tiger sharks likely seek out and exploit productive and predictable resource patches that exhibit abundant food. Tiger sharks visiting turtle rookeries or bird fledging sites are therefore no more anomalous than white sharks visiting seal rookeries. Sharks move on when the resources are depleted as some of these resources (birds, turtles) are highly seasonal. Other locations may perhaps encourage more resident behaviour, especially for pre-reproductive animals (e.g. Chesterfields/oceanic reefs), as these locations have permanent high resource abundance. Maturity/breeding may provide a powerful incentive to leave these highly productive sites.

### Reef Fidelity

Individual differences in movement patterns are not uncommon in reef-associated sharks (e.g. *C. amblyrhynchos*, [18]). Juveniles often show high site fidelity to a small region, whereas larger and older individuals are likely to move beyond a single reef or display wider ranging movements [20], [74]. To some extent, this trend remains true for the tiger shark, which, unlike smaller reef-associated shark species, shows no evidence for long-term residency in previous studies, instead exhibiting movements through large home ranges of at least 109 km [32], [35]. In our study, a SPOT track of a juvenile tiger shark in southern New Caledonia showed that this shark remained within the lagoon and close to the barrier reef (an area of approximately 3145 km^2^) (Fig. 7F), whereas four PSAT tagged sub-adult and adult tiger sharks (both male and female) migrated out of the same area and undertook wide-ranging ocean migrations. This is consistent with other studies that suggest restricted movement of young of the year (YOY) and small juvenile tiger sharks out to a depth of 100 m from the coast based on long-term catch records on the east coast of the USA [38], [75], as opposed to adults which occupy shelf and oceanic waters across the western Atlantic [1], [37]. Furthermore, the literature suggests that tiger shark movement becomes more localised over short periods (weeks) at hotspots of resource availability, such as seamounts [76], rather than in coastal areas [35], [37].

A recent review comparing horizontal and vertical movements of coastal sharks suggests fidelity is common in species that use nursery areas, but fidelity to mating, pupping, feeding and natal sites has rarely been observed [67]. Our data presents extensive fidelity to sites of tagging in the south of New Caledonia and the Chesterfields, with eight double-tagged (i.e., both satellite and internal acoustic tags) sharks detected back on our acoustic array at the site of tagging after two to 405 days (median 62 d) (Table 1). These data illustrate the potentially long-term site fidelity of large tiger sharks to specific coastal areas. Conservation of tiger sharks may be facilitated by the recently established MPAs in southern New Caledonia, especially as the southern New Caledonian coastal site may operate as a feeding area with obvious multi-year sporadic use by large tiger sharks. However, the wide ranging movements of TS 11 and other large tiger sharks also suggest a better understanding of the use of ocean habitats is necessary for effective conservation.

### Three-dimensional Habitat Use

Three-dimensional (3D) space use was estimated when the horizontal and vertical coordinates were determined simultaneously, however few studies consider 3D when describing the habitat-use of large sharks. Our study provides the first estimate of long-term 3D habitat-use by tiger sharks. Caution should be applied however, as light-based geolocation position estimates may contain considerable spatial errors compared to real time SPOT tag locations; nonetheless this method enables informed MPA design by providing an estimate of 95% of the (3D) activity space of individual tiger sharks. Clearly tiger sharks are utilising deep water habitats, which appear to be particularly important in the sub-adult and adult life history stages. MPA design for large sharks can be greatly improved if the 3D habitat use is known, particularly if incorporating open ocean areas. Our estimates of 95% home range showed large variability between individuals; however sharks frequented the epipelagic layer (0–100 m). In the vertical plane, movements are often attributed to foraging or navigation, but are less well understood than horizontal movements for almost all shark species. Hammerschlag *et al.* [37] noted that pelagic migrations by tiger sharks in the Atlantic coincide with areas of the Gulf Stream and its associated eddies that are highly productive and known for aggregations of prey including tuna and billfish. Use of deep water habitat by tiger sharks probably varies with ocean productivity, upwelling and proximity to highly productive prey patches (e.g. oceanic reefs such as the Chesterfields). Dive patterns by tiger sharks tagged in coastal areas could also be a means to utilise bathymetric cues to navigate/migrate between islands in addition to foraging [33], [61].

### Implications for Conservation and Management

The migratory movements of large tiger sharks from New Caledonia out into the Coral Sea toward Australia reflects the potential conservation implications for managing these widely separated habitats lying on a migration ‘highway’ for marine megafauna. Few fish species utilize such a remarkable range of habitat in such a short amount of time, thus tiger sharks provide novel trophic links horizontally among the shallow coastal and island reefs and open ocean as well as vertically through the epi-, meso-, and bathypelagic layers. Across the Coral Sea, tiger sharks demonstrate bi-partite habitat use (between ocean and coral reef) with high individual variability. Our data has shown direct evidence of reef site fidelity in the Chesterfield Islands, suggesting oceanic Coral Sea reefs may be particularly important for this species, both as potential mating grounds and feeding grounds for large individuals. Based on our data trends we suggest that mature females may be the primary individuals migrating between Australia and New Caledonia across the Coral Sea driven by reproductive cycles. Females may also be returning to suitable coastal areas for parturition after utilising productive ‘stop-over’ prey patches (e.g. seamounts such as the Chesterfields), hence providing important trophic links between distant reef habitats in the Coral Sea. Protection of oceanic reefs in the Coral Sea may be a critical means to conserve future stocks of this species and will require international cooperation. The conservation of tiger sharks can be facilitated in some cases by the use of coastal barrier reef marine protected areas, especially for specific sites that demonstrate continual fidelity over multiple years across individuals (such as southern New Caledonia). However these areas only provide brief protection for large life-history stages of tiger sharks which frequent pelagic waters. Oceanic migration of adults, especially females, is of particular concern. Our findings further emphasize the need to address marine conservation issues at an international scale, as top predators such as the tiger shark traverse country EEZ’s and leave the protection afforded by coastal barrier reef managed areas [11], [77]. A joint-managed (Australia and France) connectivity corridor across the Coral Sea may be one method to address this. Successful international management initiatives will, however, require more long-term research on habitat-use and migration by large tiger sharks [67]. Future research should therefore focus on comprehensive satellite tracking of mature tiger shark (both male and female) along the chain of seamounts and oceanic reefs in the centre of the Coral Sea, from the Chesterfield Islands south to LHI. Determining the role of other oceanic coral reefs should be a priority for the conservation of tiger sharks in the Coral Sea.

## Supporting Information

Video S1 **Tiger shark release.**
(MP4)

Video S2 **Juvenile tiger shark on Baited Remote Underwater Video at Lord Howe Island.**
(MP4)

## References

[1] MyersRA, BaumJK, ShepherdTD, PowersSP, PetersonCH (2007) Cascading effects of the loss of apex predatory sharks from a coastal ocean. Sci 315: 1846–1850.10.1126/science.113865717395829

[2] O’ConnellMT, ShepardTD, O’ConnellAMU, MyersRA (2007) Long-term declines in two apex predators, bull sharks (*Carcharinus leucas*) and alligator gar (*Atractosteus spatula*), in lake pontchartrain, an oligohaline estuary in southeastern Louisiana. Estuaries Coast 30 (4): 567–574.

[3] RuttenbergBI, HamiltonSL, WalshSM, DonovanMK, FriedlanderA, et al (2011) Predator-induced demographic shifts in coral reef fish assemblages. PLoS ONE 6(6): e21062.2169816510.1371/journal.pone.0021062PMC3116880

[4] DulvyNK, FreckletonRP, PoluninVC (2004) Coral reef cascades and the indirect effects of predator removal by exploitation. Ecol Lett 7 (5): 410–416.

[5] BascompteJ, MelianCJ, SalaE (2005) Interaction strength combinations and the overfishing of a marine food web. Proc Nat Aca Sc USA 102 (15): 5443–5447.10.1073/pnas.0501562102PMC55626815802468

[6] Sandin SA, Walsh SM, Jackson JBC (2010) Prey release, trophic cascades, and phase shifts in tropical nearshore marine ecosystems. In Terborgh J, Estes JA, editors. Trophic cascades: predators, prey, and the changing dynamics of nature: Island Press. 71–90.

[7] del Monte-LunaP, Lluch-BeldaD, Serviere-ZaragozaE, CarmonaR, Reyes-BonillaH, et al (2007) Marine extinctions revisited. Fish Fish 8: 107–122.

[8] Polidoro BA, Elfes CT, Sanciangco JC, Pippard H, Carpenter KE (2011) Conservation status of marine biodiversity in oceania: an analysis of marine species on the IUCN red list of threatened species. J Mar Biol: 14p.

[9] ClarkeS, Milner-GullandEJ, BjorndalT (2007) Social, economic, and regulatory drivers of the shark fin trade. Mar Res Econ 22: 305–327.

[10] Ward-PaigeCA, MoraC, LotzeHK, Pattengill-SemmensC, McClenachanL, et al (2010) Large-scale absence of sharks on reefs in the greater-Caribbean: a footprint of human pressures. PLoS ONE 5(8): e11968.2070053010.1371/journal.pone.0011968PMC2916824

[11] PalumbiSR (2004) Marine reserves and ocean neighbourhoods: the spatial scale of marine populations and their management. Annu Rev Envir Res 29: 31–68.

[12] DulvyNK, JenningsS, RogersSI, MaxwellDL (2006) Threat and decline in fishes: an indicator of marine biodiversity. Can J Fish Aquat Sci 63: 1267–1275.

[13] KnipDM, HeupelMR, SimpfendorferCA (2012) Evaluating marine protected areas for the conservation of tropical coastal sharks. Biol Cons 148: 200–209.

[14] MourierJ, PlanesS (2013) Direct genetic evidence for reproductive philopatry and associated fine-scale migrations in female blacktip reef sharks (*Carcharhinus melanopterus*) in French Polynesia. Mol Ecol 22 (1): 201–214.10.1111/mec.1210323130666

[15] PapastamatiouYP, MeyerCG, CarvalhoF, DaleJJ, HutchinsonMR, et al (2013) Telemetry and random walk models reveal complex patterns of partial migrations in a large marine predator. Ecol 94: 2595–2606.10.1890/12-2014.124400511

[16] StevensJD, BonfilR, DulvyNK, WalkerPA (2000) The effects of fishing on sharks, rays, and chimaeras (chondrichthyans), and the implications for marine ecosystems ICES J. Mar. Sci. 57: 476–494.

[17] HeupelMR, SemmensJM, HobdayAJ (2006) Automated acoustic tracking of aquatic animals: scales, design and deployment of listening station arrays. Mar Freshwat Res 57: 1–13.

[18] HeupelMR, SimpfendorferCA, FitzpatrickR (2010) Large-scale movement and fidelity of grey reef sharks. PLoS One 5: e9650.2022479310.1371/journal.pone.0009650PMC2835766

[19] BlockBA, JonsenID, JorgensenSJ, WinshipAJ, ShafferSA, et al (2011) Tracking apex marine predator movements in a dynamic ocean. Nature 475: 86–90.2169783110.1038/nature10082

[20] WerryJM, LeeSY, OtwayN, HuY, SumptonW (2011) A multi-faceted approach for quantifying the estuarine-nearshore transition in the lifecycle of the bull shark, *Carcharhinus leucas.* . Mar Freshw Res 62: 1421–1431.

[21] CluaE, SéretB (2010) Unprovoked fatal shark attack in Lifou Island (Loyalty Islands, New Caledonia, South Pacific) by a great white shark, *Carcharodon carcharias.* . Amer J Fore Med Path 31 (3): 281–286.10.1097/PAF.0b013e3181ec7cb820606572

[22] Sale PF, Cowen RK, Danilowicz BS, Jones GP, http://www.sciencedirect.com/science/article/pii/S0169534704003374 - aff4Kritzer JP, et al. http://www.sciencedirect.com/science/article/pii/S0169534704003374 - aff10(2005) Critical science gaps impede use of no-take fishery reserves. Trends Ecol Evol, 20, 74–80.10.1016/j.tree.2004.11.00716701346

[23] HammerschlagN, GallagherAJ, LazarreDM (2011) A review of shark satellite tagging studies. J Exp Mar Biol Ecol 398: 1–8.

[24] HeithausMR, HamiltonIM, WirsingAJ, DillLM (2006) Validation of a randomization procedure to assess animal habitat preferences: microhabitat use of tiger sharks in a seagrass ecosystem. J Anim Ecol 75 (3): 666–676.10.1111/j.1365-2656.2006.01087.x16689949

[25] KohlerNE, CaseyJG, TurnerPA (1998) NMFS cooperative shark tagging program, 1962–93: an atlas of shark tag and recapture data. Mar Fish Rev 60 (2): 87.

[26] FriedlanderAM, DeMartiniEE (2002) Contrasts in density, size and biomass of reef fishes between the northwestern and the main Hawaiian Islands: the effects of fishing down apex predators. Mar Ecol Prog Ser 230: 253–264.

[27] Simpfendorfer CA (2009) *Galeocerdo cuvier* (2012) IUCN red list of threatened species 2. Available: http://www.iucnredlist.org. Accessed 01 June 2013.

[28] Compagno LJV (1984) FAO species catalogue, Volume 4. sharks of the world: an annotated and illustrated catalogue of shark species known to date. Part 2. Carcharhiniformes. FAO In: Fish Synop Vol 4, parts 1 and 2. Rome: FAO. Pp. 251–655.

[29] Last PR, Stevens JD (2009) Sharks and rays of Australia. Australia CSIRO Division of Fisheries. 513 pp.

[30] LoweCG, WetherbeeBM, MeyerCG (2006) Using acoustic telemetry monitoring techniques to quantify movement patterns and site fidelity of sharks and giant trevally around French Frigate Shoals and Midway Atoll. Atoll Research Bulletin 543: 281–303.

[31] FitzpatrickR, ThumsM, BellI, MeekanMG, StevensJD, et al (2013) A comparison of the seasonal movements of tiger sharks and green turtles provides insight into Their predator-prey relationship. PLoS ONE 7(12): e51927.10.1371/journal.pone.0051927PMC352647823284819

[32] MeyerCG, ClarkTB, PapastamatiouYP, WhitneyNM, HollandKN (2009) Long-term movement patterns of tiger sharks *Galeocerdo cuvier* in Hawaii. Mar Ecol Prog Ser 381: 223–235.

[33] KohlerNE, TurnerPA (2001) Shark tagging: a review of conventional methods and studies. Environ Biol Fishes 60: 191–223.

[34] HollandKN, WetherbeeBM, LoweCG, MeyerCG (1999) Movements of tiger sharks (*Galeocerdo cuvier*) in coastal Hawaiian waters. Mar Biol 134: 665–673.

[35] HeithausMR, WirsingAJ, DillLM, HeithausLI (2007) Long-term movements of tiger sharks satellite-tagged in Shark Bay, Western Australia. Mar Biol 151: 1455–1461.

[36] MeyerCG, PapastamatiouYP, HollandKN (2010) A multiple instrument approach to quantifying the movement patterns and habitat use of tiger (*Galeocerdo cuvier*) and galapagos sharks (*Carcharhinus galapagensis*) at French Frigate Shoals, Hawaii. Mar Biol 157: 1857–1868.

[37] HammerschlagN, GallagherAJ, WesterJ, LuoJ, AultJS (2012) Don’t bite the hand that feeds: assessing ecological impacts of provisioning ecotourism on an apex marine predator. Funct Ecol 26 (3): 567–576.

[38] DriggersWB, IngramGW, GraceMA, GledhillCT, HenwoodTA, et al (2008) Pupping areas and mortality rates of young tiger sharks *Galeocerdo cuvier* in the western North Atlantic Ocean. Aquat Biol 2: 161–170.

[39] Andrews JC, http://www.sciencedirect.com/science/article/pii/019801498990037X - AFF1Clegg S (1989) http://www.sciencedirect.com/science/article/pii/019801498990037X - AFF1Coral Sea circulation and transport deduced from modal information models. Deep Sea Res Part 1 Oceanogr Res Pap. 38: 957–974.

[40] HarrisTS, HeapAD (2008) Geomorphology of the Australian margin and adjacent seafloor. Aust J Earth Sci: Int Geosci J Geol Soc Aust 55 (4): 555–585.

[41] Clua E, Gardes L, McKenna S, Vieux C (2011) Contribution to the biological inventory and resource assessment of the Chesterfield reefs. ApiaSamoa: SPREP Library. 264 p.

[42] BarnettA, AbrantesKG, SeymourJ, FitzpatrickR (2012) Residency and spatial use by reef sharks of an isolated seamount and its implications for conservation. PLoS ONE 7(5): e36574.2261578210.1371/journal.pone.0036574PMC3353940

[43] CluaE, BurayN, LegendreP, MourierJ, PlanesS (2011) Business partner or simple prey, the economic value of lemon shark in French Polynesia. Mar Fresh Res 62: 764–770.

[44] Joint statement of strategic partnership between Australia and France (2013) Available: http://www.dfat.gov.au/geo/france/joint_statement.html.Accessed 13 May 2013.

[45] OtwayNM, EllisMT (2011) Pop-up archival satellite tagging of *Carcharias taurus*: movements and depth/temperature-related use of south-east Australian waters. Mar Freshwat Res 62: 607–620.

[46] Hill RD, Braun MJ (2001) Geolocation by light level, electronic tagging and tracking in marine fisheries: proceedings of the symposium on tagging and tracking marine fish with electronic devices. East-West Center. University of Hawaii. Berlin: Springer. 315–330.

[47] LamCH, NielsenA, SibertJR (2008) Improving light and temperature based geolocation by unscented kalman filtering. Fish Res 91 (1): 15–25.

[48] R Development Core Team (2013) R: A language and environment for statistical computing. R foundation for statistical computing, Vienna, Austria. ISBN 3-900051-07-0, URL http://www.R-project.org/.

[49] Galuardi B (2010) analyzepsat. Available: http://code.google.com/p/analyzepsat/. Accessed 19 April 2013.

[50] Galuardijavascript:popRef(‘aff01’) B, François R, Golet W, Logan J, Neilson J, et al (2010) Complex migration routes of Atlantic bluefin tuna (*Thunnus thynnus*) question current population structure paradigm. Can J Fish Aqu Sci 67 (6): 966–976.

[51] NielsenA, SibertJR (2011) State–space model for light-based tracking of marine animals. Canadian J Fish Aquatic Sci. 64(8): 1055–1068.

[52] EckertSA, StewartBS (2001) Telemetry and satellite tracking of whale sharks, *Rhinocodon typus*, in the Sea of Cortez, Mexico, and the north Pacific Ocean. Env Biol Fish 60: 299–308.

[53] NakamuraI, WatanabeYY, PapastamatiouYP, SatoK, MeyerCG (2011) Yo-yo vertical movements suggest a foraging strategy for tiger sharks *Galeocerdo cuvier* Mar Ecol Prog Ser. 424: 237–246.

[54] WerryJM, LeeSY, LemckertCJ, OtwayNM (2012) Natural or artificial? habitat-use by the bull shark, *Carcharhinus leucas* . PLoS ONE 7(11): e49796.2316677210.1371/journal.pone.0049796PMC3500329

[55] CluaE, ChauvetC, ReadT, WerryJM, LeeSY (2013) Behavioural patterns of a tiger shark (*Galeocerdo cuvier*) feeding aggregation at a blue whale carcass in Prony Bay, New Caledonia. Mar Fresh Beh Physi. 46 (1): 1–20.

[56] WhitneyNM, CrowGL (2007) Reproductive biology of the tiger shark (*Galeocerdo cuvier*) in Hawaii. Mar Biol 151 (1): 63–70.

[57] BondME, BabcockEA, PikitchEK, AbercrombieDL, LambNF, et al (2012) Reef sharks exhibit site-fidelity and higher relative abundance in marine reserves on the mesoamerican barrier reef. PLoS ONE 7(3): e32983.2241296510.1371/journal.pone.0032983PMC3297616

[58] Duong T (2012) ks: Kernel smoothing. R package version 1.8.11. http://CRAN.R-project.org/package=ks. Accessed 10 April 2013.

[59] SimpfendorferCA, OlsenEM, HeupelMR, MolandE (2012) Three-dimensional kernel utilization distributions improve estimates of space use in aquatic animals. Can J Fish Aquat Sci 69: 565–572.

[60] GitzenRA, MillspaughJJ, KernohanBJ (2006) Bandwidth selection for fixed-kernel analysis of animal utilization distributions. J. Wildl. Manag 70(5): 1334–1344.

[61] Francis MP, Duffy CAJ, Bonfil R, Manning MJ (2012) The third dimension: verticle habitat use by white sharks, *Carcharodon carcharias*, in New Zealand and in oceanic and tropical waters of the Southwest Pacific Ocean. In: Domeier M, editor. Global perspectives on the biology and life history of the white shark. New York: CRC Press. 319–342.

[62] Duffy AJ, Francis MP, Manning MJ, Bonfil R (2012) Regional population connectivity, oceanic habitat, and return migration revealed by satellite tagging of white sharks, *Carcharodon carcharias*, at New Zealand aggregation sites. In: Domeier M, editor. Global perspectives on the biology and life history of the white shark. New York: CRC Press. 301–318.

[63] PatersonRA (1991) The migration of humpback whales *Megaptera novaeangliae* in east Australian waters. Mem Queensl Mus 30(2): 333–341.

[64] RevillAT, YoungJW, LansdellM (2009) Stable isotopic evidence for trophic groupings and bio-regionalization of predators and their prey in oceanic waters off eastern Australia. Mar Biol 156 (6): 1241–1253.

[65] HolmesBJ, SumptonWD, MayerDG, TibbettsIR, NeilDT, et al (2012) Declining trends in annual catch rates of the tiger shark (*Galeocerdo cuvier*) in Queensland, Australia. Fish Res. 129: 38–45.

[66] DomeierML, Nasby-LucasN (2013) Two-year migration of adult female white sharks (*Carcharodon carcharias*) reveals widely separated nursery areas and conservation concerns. Ani Biotel 1: 2.

[67] SpeedCW, FieldIC, MeekanMG, BradshawCJA (2010) Complexities of coastal shark movements and their implications for management. Mar Ecol Prog Ser 408: 275–293.

[68] Mucientes GR, Queiroz N, Sousahttp://171.66.127.192/content/5/2/156.short - aff-2 LL, Tarroso P, Sims D (2009) Sexual segregation of pelagic sharks and the potential threat from fisheries. Biol Lett 5 (2): 156–159.10.1098/rsbl.2008.0761PMC266583619324655

[69] MourierJ, VercelloniJ, PlanesS (2012) Evidence of social communities in a spatially structured network of a free-ranging shark species. Ani Beh 83 (2): 389–401.

[70] KlimleyAP (1987) The determinants of sexual segregation in the scalloped hammerhead shark *Sphyrna lewini.* Environ Biol Fish. 181: 27–40.

[71] NoriegaR, WerryJM, SumptonW, MayerD, LeeSY (2011) Trends in annual CPUE and evidence of sex and size segregation of *Sphyrna lewini*: management implications in coastal waters of north eastern Australia. Fish Res 110: 472–477.

[72] BorsaP, PandolfiM, AndréfouëtS, BretagnolleV (2010) Breeding avifauna of the Chesterfield Islands, Coral Sea: current population sizes, trends, and threats. Pac Sci 64 (2): 297–314.

[73] MatichP, HeithausMR, LayanCA (2011) Contrasting patterns of individual specialization and trophic coupling in two marine apex predators. J Ani Ecol 80 (1): 294–305.10.1111/j.1365-2656.2010.01753.x20831730

[74] GarlaRC, ChapmanDD, ShivjiMS, WetherbeeBM (2006) Movement patterns of young Caribbean reef sharks, *Carcharhinus perezi*, at Fernando de Noronha Archipelago, Brazil: the potential of marine protected areas for conservation of a nursery ground. Mar Biol 149: 189–199.

[75] NatansonLJ, CaseyJG, KohlerNE, Colket TIV (1998) Growth of the tiger shark, *Galeocerdo cuvier*, in the western North Atlantic based on tag returns and length frequencies; and a note on the effects of tagging. Fish Bull (Wash DC) 97: 944–953.

[76] Rogers AD (1993) The biology of seamounts. In: Blaxter JHS, Southward AJ, editors. Advances in marine biology, vol 30. London: Acadmic Press ltd. 305–366.

[77] MoraC, MyersRA, CollM, LibralatoS, PitcherTJ, et al (2009) Management effectiveness of the world’s marine fisheries. PLoS Biol 7(6): e1000131.1954774310.1371/journal.pbio.1000131PMC2690453

